# A distributed SDN-based intrusion detection system for IoT using optimized forests

This article has been retracted.

**DOI:** 10.1371/journal.pone.0290694

**Published:** 2023-08-30

**Authors:** Ke Luo

**Affiliations:** Fujian Vocational & Technical College of Water Conservancy & Electric Power, Fujian, China; Kebri Dehar University: Kabridahar University, ETHIOPIA

## Abstract

Along with the expansion of Internet of Things (IoT), the importance of security and intrusion detection in this network also increases, and the need for new and architecture-specific intrusion detection systems (IDS) is felt. In this article, a distributed intrusion detection system based on a software defined networking (SDN) is presented. In this method, the network structure is divided into a set of sub-networks using the SDN architecture, and intrusion detection is performed in each sub-network using a controller node. In order to detect intrusion in each sub-network, a decision tree optimized by black hole optimization (BHO) algorithm is used. Thus, the decision tree deployed in each sub-network is pruned by BHO, and the split points in its decision nodes are also determined in such a way that the accuracy of each tree in detecting sub-network attacks is maximized. The performance of the proposed method is evaluated in a simulated environment and its performance in detecting attacks using the NSLKDD and NSW-NB15 databases is examined. The results show that the proposed method can identify attacks in the NSLKDD and NSW-NB15 databases with an accuracy of 99.2% and 97.2%, respectively, which indicates an increase compared to previous methods.

## 1. Introduction

The Internet of Things (IoT) can be considered a major breakthrough in the smartification of vast networks, enabling automatic interaction among billions of heterogeneous objects [1]. This technology can be used in a wide range of applications such as smart homes, transportation systems, manufacturing industries, agriculture, and more, and its penetration rate in different fields is still increasing [2]. The reason for this can be attributed to the simplicity of the IoT concept and its significant advantages. By utilizing this technology, time, cost, and human resources can be saved, and various processes can be performed interactively and intelligently [3]. However, the use of IoT technology also comes with challenges. Security can be considered one of the most critical concerns [4]. As the IoT expands, the amount of vital information flowing through its network components also increases, and disruption in the network’s performance can lead to significant losses.

Some of the characteristics of the Internet of Things (IoT), such as its vast and heterogeneous nature, have made conventional intrusion detection strategies unsuitable for deployment in these networks [5]. This is because existing IDSs often rely on a centralized architecture for detecting attacks, which would be costly and inefficient to implement in wide-ranging IoT networks. On the other hand, existing distributed detection methods are not highly effective, and these models cannot guarantee the highest level of detection accuracy [6]. Therefore, this paper aims to address the deficiencies in IDSs for IoT structures and propose a highly accurate distributed system. The proposed method utilizes a SDN for addressing the distribution of the IDS. Furthermore, efforts are made to maximize the accuracy of the learning components used in intrusion detection through optimization techniques.

### 1.1. Research objectives, contributions and novelty

The main objective of the current research is to provide a collaborative strategy for intrusion detection in IoT and to solve some of the shortcomings of previous mechanisms to deal with attacks. This research, decomposed this goal into three minor objectives: First, introducing an efficient model for deploying detection components in the network that is compatible with the architecture of IoT. Second, using a strategy to determine the most relevant indicators with the presence of attacks on the network. Third, utilizing lightweight and accurate learning models to identify intrusions in each detection component.

The effort made to fulfill these objectives led to the formation of a novel distributed learning model named "optimized forest" that distinguishes this research from previous works. The novel contributions of this paper are as follows:

- This paper proposes a distributed architecture for IDSs based on a SDN for IoT structures. In this method, the IoT structure is divided into a set of sub-networks using SDN, and monitoring of each sub-network is assigned to a controller node. Sub-network formation is based on the positional information of objects and their movement patterns to achieve maximum stability in network communications.
- In this article, a new distributed classifier is presented, which consists of a number of optimized decision trees trained by the BHO algorithm. Each decision tree is located at a controller node and can detect the presence of attacks on the sub-networks. The decision tree deployed in each sub-network is pruned by the BHO algorithm, and the split points in its decision nodes are determined in a way that maximizes the accuracy of each tree in detecting attacks.
- The proposed IDS utilizes a collaborative strategy for decision-making regarding the presence of attacks. In this approach, participating controller nodes share their detection results and determine the existence of an attack using a majority voting strategy.

The rest of the article is organized as follows: Section two is devoted to reviewing previous relevant research in the field of intrusion detection in the IoT. In section three, the proposed method is introduced. In section four, the performance of the proposed method is evaluated from various aspects. Finally, in section five, the findings are summarized.

## 2. Related works

Due to the importance of intrusion detection in IoT networks, the number of research studies conducted in recent years regarding this issue is significant. In this section, some recent efforts to detect intrusions in IoT networks are reviewed. In [7], an anomaly-based IDS for IoT networks is presented, which utilizes deep learning techniques. This IDS uses a centralized architecture and requires monitoring all incoming and outgoing network traffic using a Convolutional Neural Network (CNN). In [8], a distributed IDS is presented to detect Distributed Denial of Service (DDoS) attacks in IoT networks. This IDS utilizes fog computing and blockchain network architecture. To this end, intrusion detection components are deployed on fog computing resources, and each component is responsible for detecting intrusions for a group of IoT devices. In this model, transactional information of fog computing resources flows through the blockchain network. Random forest and XGBoost models are also utilized for intrusion detection in the learning components.

In [9], an IDS for the IoT based on deep learning is presented. The learning model used in this IDS is a CNN. Additionally, in order to address the problem of limited training data, a Generative Adversarial Network (GAN) is utilized in this study. This neural network aims to generate artificial training samples to simulate the behavior of attacks more comprehensively based on real training samples. In [10], the focus is on the future of feature extraction and selection for intrusion detection in the IoT. In this research, a feature extraction model based on a convolutional neural network is proposed, which can transform network traffic data into a set of statistical features. Then, a feature selection model based on the Aquila (AQU) optimization algorithm is suggested, which is suitable for reducing the dimensions of features. Finally, the selected features are classified by a multi-class classifier to determine the type of attacks.

A study conducted in [11] utilizes deep learning techniques for detecting attacks in 5G networks. The proposed solution in this study includes preprocessing, feature selection, feature normalization, and detection steps. Pearson correlation criterion is used for feature selection, in which features are selected based on their correlation with the target variable (type of attacks). Additionally, detection is performed using a combination of autoencoder (AE) and Deep Neural Network (DNN). In [12], an IDS is presented for detecting attacks through IoT gateways. The detection model used in this study is a deep neural network with 5 hidden layers, which reduces the traffic features from 128 to 16 and then detects the type of attacks based on these features. In [13], an online incremental support vector data description (OI-SVDD)-based NIDS system is proposed for Industrial IoT (IIoT) devices. This NIDS system also employs adaptive sequential extreme learning machine (AS-ELM) for detecting anomalies in edge network devices.

In [14], a combination of deep learning techniques and optimization is used for intrusion detection in the IoT. In this intrusion detection model, a CNN is first utilized for feature extraction. Then, the extracted features are reduced using a feature selection algorithm based on Reptile Search Algorithm (RSA). This algorithm performs feature selection based on training error and feature correlations. Since training the model for each potential response in this algorithm would be time-consuming, determining optimal features in large datasets using this approach would be very time-consuming.

The number of studies using deep learning techniques for intrusion detection in IoT has significantly increased in recent years. For example, the model proposed in [15] introduces a lightweight convolutional neural network for use in IIoT structures. Another approach presented in [16] utilizes deep learning and transfer learning techniques for intrusion detection in IoT. Using transfer learning techniques in deep learning models can partially address the problem of labeled training data scarcity and make the deep model more efficient to train based on the small number of labeled samples. Additionally, the proposed model in [17] utilizes deep learning techniques and parallel computing for intrusion detection. The strategy used in this research involves a two-level detection system in which attack detection is performed using a signature-based model at the first level and a Cuda Long Short Term Memory Gated Recurrent Unit (cLSTM-GRU) model at the second level.

In [18], the efficient feature selection in IDSs is focused by proposing a combined feature selection algorithm called hybrid Hunger Games Search and Remora Optimization Algorithm (HHGS-ROA). The feature selection in this algorithm is based on the correlation criterion, and the selected features are classified using a Support Vector Machine (SVM). In [19], a combination of reinforcement learning and deep learning techniques is used for intrusion detection in Industrial Internet of Things. In this approach, feature selection is first performed using the LightGBM algorithm, and then the reinforcement learning-based intrusion detection agent configures the deep learning model for more efficient training.

The method proposed in [20] is a combination of optimization algorithms and machine learning for intrusion detection. In this approach, Principal Component Analysis (PCA) is used for feature extraction, and a combination of Gravitational Search Algorithm (GSA) and Differential Evolution (DE) is used to optimize the kernel function in machine learning models. In [21], a self-encoding network and Random Forests (RF) are combined to propose an IDS. Random Forests are used for feature ranking and selection, and a mixture of Gaussian model is combined with the self-encoding network for intrusion detection.

In [22], introduced an attack detection model for improving the security issues in IIoT. This security model, is a lightweight combination of Blockchain and Artificial Intelligence (AI) techniques. The AI model used in this research is a Convivial Optimized Sprinter Neural Network (COSNN), which is fed with traffic flow features. Research in [23], used combination of clustering, optimization and classification techniques to detect attacks. This research used the combination of DBScan and Anticipated Distance-based Clustering for making groups of similar data. Then Perceptual Pigeon Galvanized Optimization (PPGO) algorithm was used for parameter optimization. Finally, a Linear Naïve Bayes (LNB) classifier was used for attack detection.

Research in [24], focused on Selecting optimal features for intrusion detection in networks using evolutionary algorithms. The researchers also used SVM for classifying selected features. In [25], the application of AI techniques in IoT-based healthcare network was examined and the way of integrating these techniques with computing architectures such as cloud and edge computing was discussed. The results show the superiority of decision tree over SVM and Naïve Bayes in terms of sensitivity, precision and accuracy.

Research in [26], proposed a Blockchain-based security model for IoT which utilizes deep learning techniques for secure transmission between nodes. In [27], an edge-assisted IDS model for facing multi-attacks in IoT was introduced. This model utilized two neural networks with Back Propagation (BP) and Radial Basis Function (RBF) architectures. The BPNN model is responsible for detecting outliers and filtering flows in the first stage; while the RBFNN is used for recognition of multi-attacks in the second stage. Research in [28], introduced a security model for using in Mobile Edge Computing (MEC) environment. This model is based on managing data reputation and evaluating trust and relies on MEC devices for fast and secure processing and communication.

Research in [29], introduced deep learning-based IDS using combination of AE and SVM for IoT networks. Researchers in [30], attempted to improve the security of physical layer in IoT using Non-Orthogonal Multiple Access (NOMA) Assisted Semi-Grant-Free Transmission (SGFT). Research in [31], introduced a model named Adversarial Perturbation Against Model Stealing Attacks (APMSA), which is suitable for low cost training of deep learning models in IDSs. Researchers in [32], studied the problem of dynamic event-triggered security control in networks which are subject to packet dropouts and deception attacks. The characteristics of the works studied are summarized in Table 1.

**Table 1:** Summary of the related works.

Ref.	Year	Research Method	Advantage(s)	Disadvantage(s)
[7]	2022	anomaly-based IDS for IoT using CNN	High accuracy	Centralized architecture, High cost
[8]	2022	DDoS detection in IoT based on fog computing by RF and XGBoost	Distributed Architecture	Relatively low Accuracy, Limited to DDoS attacks
[9]	2022	IDS for IoT using CNN and GAN	Usable for small training data	High computation complexity for detection
[10]	2022	IDS for IoT using CNN and AQU optimization	Efficient reduction of dimensionality	Centralized architecture, Limited usage
[11]	2022	IDS for 5G networks using AE and DNN	High accuracy	Centralized architecture, High computation cost
[12]	2022	IDS for IoT gateways based on DNN	Low computation cost	Centralized architecture, Relatively low Accuracy
[13]	2022	NIDS for IIoT based on OI-SVDD and AS-ELM	Distributed Architecture	Limited usage
[14]	2022	IDS for IoT using CNN and RSA	High accuracy	High computation complexity for detection
[15]	2022	IDS for IIoT based on lightweight CNN	Low computation cost	Centralized architecture, Lack of generality
[16]	2022	IDS for IoT using CNN and transfer learning	Usable for small training data	High computation complexity, Centralized
[17]	2022	Two-step IDS for IoT using signature analysis and cLSTM-GRU	High accuracy	High computation complexity, Limited to hardware, Centralized
[18]	2022	IDS for IoT using HHGS-ROA and SVM	Efficient reduction of dimensionality	Centralized architecture
[19]	2022	IDS model using LightGBM and deep reinforcement learning	Efficient training of model by reinforcement learning	High computation complexity, Centralized
[20]	2020	IDS for IoT using PCA and GSA-DE	Usable for unbalanced and small training data	Inefficient feature extraction, Centralized
[21]	2020	IDS model based on self-encoding network and RF	Low computation cost	Centralized architecture, Relatively low Accuracy
Proposed Work		A distributed SDN-based IDS model for IoT using combination of BHO and decision trees		

## 3. Proposed model

An IDS for the IoT should not only use an accurate model for detecting attacks but also use an efficient architecture to reduce monitoring costs. To this end, a distributed, SDN architecture is used in the proposed method. The proposed method also uses a set of optimized decision trees generated by the BHO Algorithm as its learning model for intrusion detection. The proposed method consists of the following main phases:

1. Network partitioning and deployment of learning models for intrusion detection.
2. Optimized forest-based intrusion detection.

The structure of the proposed method is shown in Fig 1. Note that the first phase is applied globally to the entire network, while the second phase is executed independently on each sub-network obtained in the first phase. In the first phase, the network structure is partitioned into a set of sub-networks, and monitoring of each sub-network is assigned to a controller node. The aim of this is to improve the distributability of the proposed model and reduce the costs of monitoring network traffic. Each monitoring controller uses a decision tree-based learning model to detect attacks. These learning models can perform the intrusion detection process independently or collaboratively, and these processes are explained in detail in the second phase of the proposed method. Since each decision tree model is optimized independently using the Black Hole Algorithm, the set of learning models used in the proposed IDS is referred to as an optimized forest. In general, the intrusion detection process in the second phase consists of “preprocessing”, “feature selection”, “tree optimization”, and “classification” steps. The rest of this section explains the details of each phase in the proposed method. Also, the table of notations used in this section is presented in Table 2.

**Fig 1:** The structure of the proposed method.

**Table 2:** The table of notations.

Symbol	Description
*T*_*i*.*j*_	Durability of the communication between nodes I and j
*v*_*ij*_	Relative velocity between nodes i and j
*φ*_*ij*_	Relative angle between nodes i and j
*v*_*i*_	Velocity of node i
*φ*_*j*_	Direction of motion in node j
*Δt*	Threshold of communication durability between each pair of neighbor nodes
*N*_*F*_	Normalized vector of feature F
*H*(*X*)	Entropy of feature set X
*p*_*X*_(*f*)	The ratio of the elements in f to the number of elements in X
*X*_*BH*_	The position of black hole in BHO algorithm
*X*_*i*_	The position of star i in BHO algorithm
*f*_*BH*_	The fitness of the black hole in BHO algorithm
NP	The number of stars in the population of BHO algorithm
N	Number of decision nodes in initial decision tree to be optimized
M	Number of leaf nodes in initial decision tree to be optimized

### 3.1. Network partitioning and deployment of learning models for intrusion detection

In the first phase of the proposed method, the network structure is decomposed into a set of sub-networks, and the task of monitoring each sub-network is assigned to a controller node. To do this, the list of neighbors of each active node in the network must first be identified, which is done by exchanging Hello control packets. In this process, each node stores its unique ID in the content of the control packet and then, by broadcasting this message, notifies its existence to its neighboring nodes. Upon receiving this message, each active node will add the sender’s node ID to its list of neighbors. By repeating this process, each active node will produce a list containing its neighbor’s IDs. Then, each active node in the network will send its properties, including its ID, location information, neighbor list, and radio communication range, to the central SDN controller through a control packet. After receiving all control packets by the central controller node, it will create a view of the communication pattern of the network nodes, and it will be able to create the adjacency graph of the active nodes in the network. Based on the received location information, the central SDN controller can calculate the durability of the communication between each pair of neighboring nodes [33]:

$$T_{i.j}=\frac{d.cos(\varphi_{ij})+\sqrt{r^{2}-d^{2}\sin^{2}\left(\varphi_{ij}\right)}]}{v_{ij}}$$ (1)

$$v_{ij}=\sqrt{{\left(v_{i}\;\cos\left(\varphi_{i}\right)-v_{j}\;\cos\left(\varphi_{j}\right)\right)}^{2}+{\left(v_{i}\;\sin\left(\varphi_{i}\right)-v_{j}\;\sin\left(\varphi_{j}\right)\right)}^{2}}$$

$$\varphi_{ij}=\tan^{-1}\frac{v_{i}\;\sin\left(\varphi_{i}\right)-v_{j}\;\sin\left(\varphi_{j}\right)}{v_{i}\;\cos\left(\varphi_{i}\right)-v_{j}\;\cos\left(\varphi_{j}\right)}$$

The above equation shows that *v*_*i*_ represents the speed of node i and *φ*_*i*_ determines its direction of motion. Also, r represents the radio communication range of the node, and d represents the distance between nodes i and j, which is estimated by sampling the received signal strength indicator (RSSI). Using the above equations, the approximate time that nodes i and j will remain neighbors can be calculated. By calculating the value of *T*_*i*.*j*_ for each pair of nodes in the network, a similarity matrix is formed. This matrix contains the similarity of the motion pattern of each pair of nodes. The central SDN controller, in order to decompose the network into a set of subnets, uses two basic rules:

- Each pair of nodes located in a subnet must have each other in their neighborhood list.
- The duration of the connection between two nodes belonging to a subnet should be greater than a time threshold *Δt* (*T*_*i*,*j*_≥*Δt*).

Based on these rules, the stages of network decomposition by the central controller node will be as follows:

Algorithm 1: SDN-based network partitioning

*Input*: A list of network nodes L, a connectivity matrix T

*Output*: Object categories of the network C

1. Repeat the following steps until a node is in the list L:

2. Choose a random node x from the list L and remove it from L. Create a new cluster in C.

3. For each node y ∈ L, if y is a neighbor of x and based on matrix T, we have *T*_*x*.*y*_≥*Δt*, then add y to the current category in C and remove node y from list L.

4. If *L* = *ϕ*, go to the next step, otherwise repeat from step 1.

5. Return the clusters C as the output.

After performing this step, all nodes in the network are places into clusters corresponding to their movement pattern. Then, each group of objects in clusters C is considered as a sub-network. The central SDN controller assigns a controller node to each of the formed sub-networks, whose task is to monitor the input and output traffic of that sub-network. The process of monitoring sub-networks and detecting attacks is performed using an optimal decision tree model deployed on the controller of that sub-network. Each controller node can perform the intrusion detection process independently or collaborate with other controller nodes and perform this action through voting techniques. These processes are described in the next section.

### 3.2. Intrusion detection in each sub-network based on optimized forest

Each controller supervising the sub-networks formed in the first phase of the proposed method uses an optimized decision tree generated by BHO algorithm to detect attacks. Thus, the input and output traffic of the sub-network is analyzed and the presence of attacks is examined using this model. However, accurate differentiation of normal network activities from attacks, data preparation, and the use of appropriate features are necessary to perform the detection process by the learning model with the highest accuracy. Therefore, the intrusion detection process in each sub-network is performed through the following partial steps:

1. preprocessing
2. Feature selection
3. Constructing and optimizing decision tree model
4. Detection

The goal of preprocessing is to prepare input data in a way that necessary computational processes for detecting attacks can be performed on them. In the second step, a subset of input features is selected using Analysis of variance (ANOVA) and sequential feature selection (SFS) technique. The aim of this step is to remove redundant information and achieve more accurate intrusion detection with minimal necessary information. To detect intrusion in each sub-network, a decision tree is used, the structure of which is optimized using the BHO algorithm in the third step. Finally, the optimized learning model is used for detecting attacks.

#### 3.2.1. Preprocessing

The first step in the proposed IDS is to prepare the data through preprocessing. In the proposed method, data preprocessing starts with managing missing values. To do so, all training records with missing values are ignored. After this step, nominal features are converted to numeric ones. This is done separately for each feature. First, the unique nominal values of each feature are extracted and then these values are sorted in ascending order based on their frequency in the training records. Finally, a natural number is assigned to each nominal value based on the obtained order, and the assigned number is used to replace the nominal values. By performing these operations, data records are converted to a set of numeric features. The preprocessing step ends with mapping the feature values to the range [0,1]. This is done for each feature, such as F, using the following equation [34]:

$$N_{F}=\frac{F-min_{F}}{max_{F}-min_{F}}$$ (2)

In the above equation, *min*_*F*_ and *max*_*F*_ denote the minimum and maximum values in the feature vector F, and *N*_*F*_ describes the corresponding normalized vector of F.

#### 3.2.2. Feature selection

In the second step of the proposed intrusion detection method, feature selection is performed using a simple yet effective strategy that selects a subset of features that is close to optimal with minimal computational cost. This is done using ANOVA and the SFS strategy [35].

First, the F-score of the input features is calculated using a one-way ANOVA test. This provides a numerical score that describes the importance of each feature. Generally, features with high F-scores are more important, and reducing their scores decreases their importance. Therefore, the input features are sorted in descending order based on their F-scores, with the most important feature at the beginning of the list and the least important feature at the end.

The next step in feature selection is to determine the number of features that can achieve the highest detection accuracy. The SFS strategy is used to achieve this goal. In this strategy, the first two features with the highest F-scores are added to the selected features list, and a decision tree model is constructed based on these features. Then, the training error of the created tree is calculated.

In a repetitive process, a new feature with the highest F-score is added to the selected features set, and the process of constructing the decision tree and calculating the training error is repeated. If the training error decreases, the process of adding new features based on their F-scores is repeated. However, if adding a feature increases the training error (decreases accuracy), the algorithm terminates, and the feature list with the lowest training error is considered the selected features.

This feature selection process reduces the number of input features while maintaining the detection accuracy of the model. The selected features are used as inputs for the next step of the intrusion detection process.

#### 3.2.3. Constructing and optimizing decision tree model

In each controller node, which supervises the sub-networks formed in the first phase of the proposed method, a decision tree is used to detect intrusion. Existing algorithms for building decision trees cannot guarantee achieving the optimal tree. For this reason, in this step, the BHO algorithm is used to optimize the structure of a decision tree.

It should be noted that in the proposed method, the process of building and optimizing trees is done independently in each controller node, and thus, the decision tree structures created in each controller can be different from others. The basic decision tree structure used in the proposed IDS is C4.5. Therefore, first, an initial decision tree is created in each control node based on the C4.5 decision tree building algorithm, and then, the structure of this tree is optimized using the BHO algorithm.

The optimization of the decision tree structure in the proposed method includes pruning the tree and adjusting the split points in its decision nodes. In each decision tree, nodes are divided into two categories of decision nodes and leaf nodes. Each decision node includes two branches, and based on them, classification rules for samples can be followed based on the values of their features. On the other hand, leaf nodes determine the end points of the decision tree, and based on them, it can be determined in which of the target classes each sample belongs. The basic decision tree building algorithm in the proposed model is based on the approach presented in [36]. This method uses the information gain (IG) measure to build the tree [36]:

$$IG(X.Y)=H(X)-\sum_{f\in F}p_{X}(f)H(f)$$ (3)

Where H(X) represents the entropy of set X, and F determines the subsets generated by dividing set X using feature Y, such that we have: *X* = ∪_*f*∈*F*_*f*. Also, *p*_*X*_(*f*) represents the ratio of the number of elements in f to the number of elements in set X. In the process of building the basic tree, first the information gain of each feature is calculated from the input data set X, and then the set X is divided into subsets using the feature that has the most information gain. Then, a decision node for the selected feature is added to the tree structure, and according to the remaining features, this operation is repeated on the subsets created for X in a recursive manner. During the recursive process of tree construction, if all the examples of the subset belong to the same class; a leaf node will be created.

In the following, the mechanism of optimizing constructed tree by BHO algorithm is described. BHO, is nature-inspired optimization algorithm which tries to solve problems by modeling the motion pattern of stars and black holes. BHO is a population-based algorithm whose characteristics such as the simplicity of the mechanism and effective search of the problem space have made it possible to use it in solving different problems. In this algorithm, each candidate solution is considered as a star and the best solution is modeled as a black hole. BHO, initiates with constructing a random population of stars in the search space. Then, the fitness of each star is evaluated and a star with the best position in the population is considered as a black hole. After determining the black hole in the current population, the position of each star is updated as follows [37]:

$$X_{i}=X_{i}+rand.(X_{BH}-X_{i})$$ (4)

Where, *X*_*BH*_ represents the position of black hole and *X*_*i*_ denotes the position of star *i*. This operation, makes the stars to search the problem space for better solutions. A black hole can absorb the stars located around it. To model this behavior, BHO uses a radius threshold value which is calculated as follows [37]:

$$R=\frac{f_{BH}}{\sum_{i=1}^{NP}f_{i}}$$ (5)

Where, *f*_*BH*_ and *f*_*i*_ represent the fitness of the black hole and the fitness of star i, respectively,. Also, NP determines the number of stars in the population of optimization algorithm. Therefore, after updating the position of stars, their distance with black hole is measured. If a star is in the radius R of the black hole; Then that star is swallowed by the black hole and a new star is randomly created in the problem space. This mechanism can effectively prevent candidate solutions from being trapped in local optima. Next, based on an iterative process, the new position of black hole is determined and the processes of updating the position of the stars and being swallowed by the black hole are repeated. This process is repeated until the termination conditions of the algorithm are met.

The optimization problem discussed in this phase of the proposed method is adjusting the split points in decision nodes and pruning the created tree. Therefore, for a basic decision tree with N decision nodes and M leaf nodes, the optimization variables in this problem can be divided into two categories:

- N real variables, each corresponding to one of the decision nodes in the tree and its value indicating the division point in that node. Since all input variables of the problem are normalized using Eq (2), the search bounds for all these variables will be (0, 1).
- M binary variables, each corresponding to one of the leaf nodes in the tree. In these variables, the value of zero means pruning the branch corresponding to that leaf node in the tree structure, while the value of one indicates keeping that node in the tree structure.

Considering the set of the above variables, each solution vector (star) in the proposed BHO algorithm for optimizing the decision tree will have a heterogeneous structure consisting of *N*+*M* elements. In each solution vector, the first N elements are used to determine the split points of decision nodes, while the last M elements specify the removal or retention of leaf nodes in the tree structure.

Fig 2 shows examples of solution vector structures. A basic decision tree is shown in Fig 2A. Since the assumed tree consists of four decision nodes (*D*_1_.*D*_2_.*D*_3_.*D*_4_) and five leaf nodes (*A*.*B*.*C*.*D*.*E*), the length of each solution vector for optimizing this tree in the optimization algorithm will be 9, in which the real values in the first four elements are used to determine the split points of the tree and the values in the next five binary elements are used for pruning the leaf nodes of the tree. Fig 2B shows a hypothetical solution vector structure for editing this tree. Applying this solution vector on the assumed basic tree will result in the tree shown in Fig 2C. For example, the second element of this solution vector specifies the split point determined for the decision node *D*_2_, which is assigned a value of 0.05, and based on this value, the corresponding condition for this decision node is set to *D*_2_>0.05. Since the decision tree structure used in the proposed method is binary, by removing one of the children of a decision node, the remaining leaf node replaces the mentioned decision node. For example, by removing the leaf node E (which is the child of the decision node *D*_4_), the node *D*_4_ will be converted into a leaf node labeled D. The result of the pruning process for the assumed tree is shown in Fig 2D.

**Fig 2:** A sample solution vector and how to apply it to the basic decision tree for optimization in the proposed method.

After applying each vector to the original tree structure, the fitness of solution vector can be calculated based on the obtained tree. In the proposed method, the training error criterion is used as the fitness function in the BHO algorithm. To do so, the training samples are applied to the tree corresponding to the solution vector, and the output labels obtained from the tree are compared with their true labels for these samples. Then, the fitness of solution vector can be calculated as follows:

$$f_{x}=\frac{E}{T}$$ (6)

Where E represents the number of training samples for which the tree output is different from their true label and T represents the total number of training samples. Thus, by using the proposed structure for the solution vector, decision nodes in the learning model can be efficiently adjusted while pruning the tree. Using the training error criterion as the fitness function in the proposed optimization algorithm guarantees achieving the minimum prediction error in the obtained learning model. Since the initial population of solution vectors in the BHO algorithm is based on the C4.5 model at the beginning of this phase, it can be concluded that the optimized model using the proposed method will have a minimum accuracy equal to the base C4.5 model. Considering the described structure for the solution vector and the fitness function, the steps for optimizing decision tree by the BHO algorithm will be as follows:

Algorithm 2: Optimizing trees by BHO

*Step 1*: The initial population of solution vectors is randomly determined based on the specified optimization variables.

*Step 2*: Fitness of each solution vector is calculated using Eq (6).

*Step 3*: The star (solution) with the minimum fitness is considered as a black hole denoted as *X*_*BH*_.

*Step 4*: The position of each star is updated using Eq (4).

*Step 5*: The threshold distance R of black hole is calculated using Eq (5).

*Step 6*: If a star like *X*_*i*_ has a fitness less than the fitness of *X*_*BH*_, then set *X*_*BH*_ = *X*_*i*_ and *f*_*BH*_ = *f*_*i*_.

*Step 7*: If the distance of a star like *X*_*i*_ to the black hole is less than the threshold R (*X*_*i*_−*X*_*BH*_≤*R*), then randomly generate the position of *X*_*i*_ in the problem space.

*Step 8*: Terminate the algorithm if one of the termination conditions is met, otherwise go to Step 2.

Based on the above steps, the basic decision tree structure will be optimized. The termination conditions of the BHO algorithm in proposed method include:

- One of the solutions in the population reaches zero fitness.
- The number of iterations of the algorithm reaches the threshold T.

#### 4.2.3. Intrusion detection

The final step in the intrusion detection phase in the proposed method is the classification of information using decision tree models located in the controller nodes. As mentioned, each controller node can independently perform intrusion detection or perform it through collaboration with other controller nodes. The intrusion detection pattern can be determined based on network conditions by the designer. If a controller node performs intrusion detection independently, it will examine all incoming and outgoing traffic through its sub-network before routing, using the optimal decision tree located in its memory. If the decision tree’s result indicates an attack, the input/output connection for that flow will be aborted; otherwise, incoming/outgoing traffic will flow normally. Conversely, if the collaborative strategy is used for intrusion detection in the controller nodes, all participating controller nodes in the traffic flow will first analyze traffic flow features and share their local detection results with other controller nodes. Then, using the majority voting strategy, they determine the final result for detecting the presence of an attack. If the voting result indicates an attack’s presence, all the mentioned controller nodes cancel the connection. Although the use of the collaborative strategy increases the communication overhead of the network in the intrusion detection process, it has two significant advantages. First, the use of the collaborative strategy enables the combination of the learning ability of multiple models in the intrusion detection process, achieving higher detection accuracy. Because by using multiple learning models simultaneously, errors in some learning models can be covered. The second advantage of using a collaborative strategy for intrusion detection is providing a higher level of network security and preventing the infection of intermediate devices. An example of this process is shown in Fig 3.

**Fig 3:** Examples of collaborative (top) and independent (bottom) intrusion detection processes in controller nodes by the proposed method.

In the upper part of Fig 3, an example of a cooperative strategy for intrusion detection is given, in which three controller nodes C_1_, C_2_ and C_3_ cooperate to detect a possible attack in the traffic flow between two nodes x and y. It is assumed that the result of local detection of controller nodes C_1_, C_2_ and C_3_ is "normal", "attack" and "attack" respectively. By voting between the detection results of these three controller nodes, the result of aggregation will be "attack". As a result, communication between two nodes x and y is prevented. As shown, this process avoids forwarding data and possible contamination of the C_2_ subnet. The results related to the independent detection mode of the controller nodes are illustrated in the bottom part of Fig 3. Since the learning model based on the controller C_1_ has not been able to detect the attack, it forwards the malicious traffic flow to the intermediate subnet C_2_.

## 4. Simulation and results

The proposed method has been implemented using MATLAB 2020a software. In the simulation environment, an IoT-based network consisting of 500 nodes with heterogeneous characteristics was considered, and 10% of the objects have mobility in the environment. The simulation environment dimensions are set to 200m×200m. During the experiments, data from two databases, NSLKDD [38] and NSW-NB15 [39], were used to simulate node behavior. Next, we will first explain the characteristics of these two databases and then discuss the results obtained from the experiments.

### 4.1. Database and evaluation metrics

The first database used to evaluate the performance of the proposed method is NSLKDD. This database was presented to address the deficiencies of the KDD’99 database and has a similar structure to it. In this database, each record contains traffic information obtained from communications between node pairs, described using 41 features. The initial number of samples in this database is 1074992, of which a significant portion is repetitive, and the number of unique records is approximately 126000. Due to the large number of samples, 20% of the data from this database, consisting of 25192 data records, has been used in these experiments. The class of each data record is identified by a nominal label. In the dataset used, 13413 samples belong to the normal class, and the rest indicate the presence of an attack.

The second database used is the NSW-NB15 dataset, which includes newer types of attacks and resolves the shortcomings of older databases such as KDD99 or NSLKDD. The number of samples in this database is 2540044. Each data record is described by 49 attributes, which include packet-based and flow-based attributes. In general, the attributes of this database can be divided into four categories: packet header-based features, time features, flow features and content features. The number of classes in this database is equal to 10 (normal and 9 types of attacks). About 87.35% of the samples of this database belong to the normal class. Due to the high number of samples and also the high asymmetry in the samples of each category, 80% of the samples belonging to the normal class in the NSW-NB15 database have been ignored. By doing this, the number of samples in the database was reduced to 508,000, in which 186,717 samples belong to the normal class and the rest of the samples indicate the existence of an attack.

In order to evaluate the proposed method, the simulation process was repeated 10 times. In each repetition, 90% of the samples were used to train the learning models and the remaining 10% were used as traffic features generated by network objects (test samples). Each test sample was used only once, and after 10 repetitions of the experiment, all data samples were labeled using the proposed method. During the experiments, the intrusion detection problem was considered as a binary classification problem, where the samples related to normal traffic were considered as negative class and the types of attacks were considered as positive class. After classifying each sample by the learning model, the predicted label was compared with the actual label of the sample, and the classification result was determined in one of the following cases:

- TP: occurs when an attack is correctly classified by the learning algorithm.
- TN: relates to the conditions where a normal sample is correctly labeled.
- FP: occurs in cases where a normal sample is mistakenly identified as an attack.
- FN: relates to the case where an attack is wrongly classified as a normal sample.

Based on these cases, accuracy, precision, recall, and F1 metrics were used to evaluate the performance of the proposed method in detecting attacks. The accuracy metric indicates the ability of the model to detect intrusions in correctly distinguishing normal and attack samples and is calculated as follows:

$$Accuracy=\frac{TP+TN}{TP+TN+FP+FN}$$ (7)

The precision metric indicates the probability that the detected attacks by the IDS are correct and is calculated as follows:

$$Precision=\frac{TP}{TP+FP}$$ (8)

The recall metric indicates the proportion of all attacks that the IDS was able to identify:

$$Recall=\frac{TP}{TP+FN}$$ (9)

Finally, the F1 metric is the harmonic mean of precision and recall metrics, which is calculated as a weighted value based on these two metrics, and based on that, the performance of the proposed method can be evaluated.


$$F1=\frac{2\times Precision\times Recall}{Precision+Recall}$$ (10)

### 4.2. Results and discussion

Based on the data and configuration described in the previous section, the performance of the proposed method was evaluated. During the experiments, the population size and number of iterations in the BHO algorithm were set to 200 and 300, respectively, to optimize the decision tree structures. The performance of the proposed method was evaluated in two modes of “collaborative detection by controller nodes” and “independent detection”. Additionally, to examine the effectiveness of the decision tree optimization strategy using the BHO algorithm, the results of the proposed method were compared with a baseline method that uses the C4.5 decision tree without optimization for intrusion detection. Fig 4 illustrates the average accuracy of the proposed method in detecting attacks for the NSLKDD and NSW-NB15 datasets compared to other methods.

**Fig 4:** The average accuracy of the proposed method in detecting attacks through (a) NSLKDD and (b) NSW-NB15 databases.

Based on the charts presented in Fig 3, the proposed method can detect attacks with higher accuracy than the compared methods for both datasets used in the experiments. According to these results, using a collaborative strategy for intrusion detection in the proposed method will have the highest accuracy in both evaluated datasets. However, it is still possible to improve the detection accuracy by using the intrusion detection strategy independently by the controller nodes. The analyses show that the collaborative strategy can increase the detection accuracy by 0.263% and 0.85% in NSLKDD and NSW-NB15 databases, respectively, compared to the independent detection strategy. On the other hand, comparing the proposed model (optimized decision tree using the BHO algorithm) with the basic C4.5 model indicates that the proposed optimization strategy can increase the accuracy of decision tree models by 3.04% compared to conventional models. This difference in classification accuracy demonstrates the effectiveness of the proposed optimization strategy in adjusting the splitting point of decision nodes and pruning the tree. In Fig 5, the confusion matrix for various algorithms for detecting attacks in the NSLKDD dataset is presented.

**Fig 5:** Confusion matrix resulting from detection of attacks in the NSLKDD database by different methods.

In Fig 5A, the confusion matrix for the proposed method in the collaborative detection mode is shown. In these matrices, labels 1 and 2 indicate negative (normal traffic) and positive (attacks) classes, respectively. Also, the rows of these matrices represent the predicted labels by each method, while the columns represent the ground truth labels. Therefore, the proposed method correctly classified 13,312 test samples from the negative category (TN), and only misclassified 101 test samples from this category as positive (FP). On the other hand, out of 11,779 positive test samples, the proposed method correctly classified 11,672 test samples as positive (TP), but it also misclassified 1,107 test samples from this category as negative (FN). In this way, the proposed method had an error in classifying only 208 samples out of the total samples of the NSLKDD data set, which resulted in an accuracy of about 99.2% of the proposed method. Based on these results, the performance of the proposed method is equal to 99.1 and 99.2 percent in terms of sensitivity and specificity criteria. Comparing the confusion matrix of the proposed method with other methods shows that the solution proposed in this research has a better performance for detecting attacks in NSLKDD dataset samples. Based on these results, the method presented by Saba et al. in [7] has the closest performance to the proposed method and was able to correctly classify 98.9% of the samples. Based on these results, the sensitivity and specificity of this method is equal to 98.9%. The confusion matrix of different algorithms for detecting attacks in the NSW-NB15 dataset is shown in Fig 6.

**Fig 6:** Confusion matrix resulting from detection of attacks in the NSW-NB15 database by different methods.

The comparison of the matrices shown in Fig 6 demonstrates that the proposed method also outperforms the compared methods in the NSW-NB15 dataset. Accordingly, the sensitivity and specificity of the proposed method (in collaborative detection mode) for the NSW-NB15 dataset are 97.2%, which represents a 1.1% improvement compared to the closest method. Therefore, the proposed method has superiority in correctly classifying both positive and negative samples compared to the compared methods.

In Fig 7, various intrusion detection methods are compared in terms of accuracy, recall, and F-measure for the NSLKDD and NSW-NB15 datasets. The results presented in Fig 7 confirm that the proposed method can detect attacks in both datasets with higher efficiency. The higher accuracy of the proposed method means that the detection outputs as attacks have a higher probability of being correct. On the other hand, the higher recall score indicates that the proposed method can correctly classify a higher percentage of attacks. The performance superiority of the proposed method can be attributed to the use of the BHO algorithm for optimizing decision tree models. Additionally, the collaborative strategy for intrusion detection enables the combination of the capabilities of several learning models for detecting attacks, thus reducing the probability of error occurrence.

**Fig 7:** Classification quality for (a) NSLKDD dataset and (b) NSW-NB15 dataset by different methods.

In Fig 8, the Receiver Operating Characteristics (ROC) curve obtained from the classification of samples from the two datasets used for different methods is shown. To better display performance differences between methods, the display range of the curve has been zoomed in Fig 8A.

**Fig 8:** ROC curve resulting from the classification of samples of (a) NSLKDD dataset and (b) NSW-NB15 dataset.

Based on the plotted graphs in Fig 8, the proposed method has higher true positive rates and lower false positive rates, and its area under ROC curve is greater than the compared methods. Therefore, it can be concluded that the proposed method in this article has a higher average accuracy in correctly classifying attacks. The numerical values of the experiments conducted in this article are presented in Table 3.

**Table 3:** The numerical values of the experiment results.

Database	Method	Accuracy	F-measure	Recall	precision
**NSLKDD**	Proposed (Cooperative)	99.1743	99.1708	99.1693	99.1724
	Proposed (Individual)	98.9124	98.9078	98.9114	98.9044
	C4.5	98.0113	98.0031	98.0083	97.9980
	Saba et al [7]	98.8885	98.8839	98.8869	98.8809
	Fatani et al [10]	98.6623	98.6569	98.6667	98.6476
**NSW-NB15**	Proposed (Cooperative)	97.1654	96.9645	97.1702	96.7728
	Proposed (Individual)	96.3154	96.0591	96.3193	95.8218
	C4.5	94.1213	93.7306	94.1130	93.4008
	Saba et al [7]	96.0921	95.8220	96.0998	95.5704
	Fatani et al [10]	95.1256	94.7958	95.1330	94.4983

Based on the results presented in Table 3, the proposed method can detect attacks with higher efficiency in terms of various criteria. These results demonstrate the effectiveness of the proposed strategy in real-world scenarios.

### 4.3. Limitations and future works

The proposed method used SDN as an infrastructure for deploying the IDS model. This is while the SDN architecture itself has security issues that need to be addressed. For example, the biggest security issue about SDN is the communication channel. Because, the Open Flow protocol, uses Transport Layer Security (TLS) for data-control channel communication security, and it is prone to Man-In-The-Middle (MITM) attacks. Addressing these issues requires the use of security strategies that are outside the scope of this research; But solving them in order to guarantee the performance of SDN-based IDSs is of great importance. For this reason, solving the security issues related to the communication channel in SDN can be a topic for continuing this research path.

As the IDS proposed employs a set of decision tree models for intrusion detection, and these tree models are formed based on rules extracted from past observations, it cannot be certain about its performance in detecting new and unknown attacks. To overcome this limitation in the proposed method, decision tree models can be combined with fuzzy inference models to enhance the flexibility of the model in detecting unknown attacks. On the other hand, optimizing the decision tree model using the BHO algorithm in the proposed method increases the computational load of the system during the model training phase. Although this increase in computation only occurs during the training phase, the time difference can be minimized using parallel processing techniques.

## 5. Conclusion

Security and intrusion detection are one of the most important challenges in large computer networks such as the Internet of Things. With the development of computing technologies, intrusion techniques have also advanced, leading to an increasing need for more efficient systems to detect attacks. In this article, a distributed method for detecting intrusions in IoT networks is presented. The proposed method consists of two phases, network decomposition and intrusion detection. In the first phase, the network structure is divided into a set of sub-networks using SDN. The aim of this is to improve the distributability of the proposed model and reduce the cost of network traffic monitoring. To this end, each sub-network is monitored by a controller node in the proposed method. Each controller node uses a decision tree-based learning model to detect attacks in its sub-network. The decision tree deployed in each sub-network is pruned by the BHO algorithm, and the split point of its decision nodes are also determined in a way that maximizes the accuracy of each decision tree in detecting attacks. The proposed architecture also uses a collaborative strategy for decision making regarding the existence of attacks. In this method, participating controller nodes share their detection results and determine the presence of an attack using a majority voting strategy. The use of this technique can increase the accuracy of attack detection compared to previous strategies. The performance of the proposed method was evaluated using two NSLKDD and NSW-NB15 databases. During the experiments, accuracy, precision, recall and F-Measure criteria were used to fully study the proposed IDS. The results showed that the optimization of the decision tree structure by the BHO algorithm in the proposed method can increase the accuracy of attack detection by 3.04%. On the other hand, the proposed collaborative strategy based on majority voting can be effective in increasing the accuracy percentage from 0.26 (for NSLKDD dataset) to 0.85 (for NSW-NB15 dataset). These results showed that the proposed method can detect the presence of attacks in the NSLKDD and NSW-NB15 databases with an average accuracy of 99.2 and 97.2%, which is an improvement compared to previous methods.
